# Comparative Effects of Retinoic Acid or Glycolic Acid Vehiculated in Different Topical Formulations

**DOI:** 10.1155/2015/650316

**Published:** 2015-01-06

**Authors:** Patrícia Maria Berardo Gonçalves Maia Campos, Lorena Rigo Gaspar, Gisele Mara Silva Gonçalves, Lúcia Helena Terenciane Rodrigues Pereira, Marisa Semprini, Ruberval Armando Lopes

**Affiliations:** ^1^Faculdade de Ciências Farmacêuticas de Ribeirão Preto, Universidade de São Paulo, Avenida do Café, s/n, 14040-903 Ribeirão Preto, SP, Brazil; ^2^Faculdade de Ciências Farmacêuticas, Pontifícia Universidade Católica de Campinas, 13060-904 Campinas, SP, Brazil; ^3^Faculdade de Odontologia de Ribeirão Preto, Universidade de São Paulo, 14040-904 Ribeirão Preto, SP, Brazil

## Abstract

Retinoids and hydroxy acids have been widely used due to their effects in the regulation of growth and in the differentiation of epithelial cells. However, besides their similar indication, they have different mechanisms of action and thus they may have different effects on the skin; in addition, since the topical formulation efficiency depends on vehicle characteristics, the ingredients of the formulation could alter their effects. Thus the objective of this study was to compare the effects of retinoic acid (RA) and glycolic acid (GA) treatment on the hairless mouse epidermis thickness and horny layer renewal when added in gel, gel cream, or cream formulations. For this, gel, gel cream, and cream formulations (with or without 6% GA or 0.05% RA) were applied in the dorsum of hairless mice, once a day for seven days. After that, the skin was analyzed by histopathologic, morphometric, and stereologic techniques. It was observed that the effects of RA occurred independently from the vehicle, while GA had better results when added in the gel cream and cream. Retinoic acid was more effective when compared to glycolic acid, mainly in the cell renewal and the exfoliation process because it decreased the horny layer thickness.

## 1. Introduction

Retinoids and hydroxy acids have been widely used in cosmetic products and in dermatology to revert the photoageing process and superficial wrinkles and also in the acne treatment [1–3]. In addition, these substances have been used in chemical peels for the treatment of skin aging, particularly photodamage [4–6].

Retinoic acid is used at 0.025%, 0.05%, and 0.1% concentrations for acne and photoageing treatment. The mechanism of action of retinoids has not been completely elucidated, but these substances could have profound effects on the modulation of cellular proliferation and differentiation. These effects are known to be mediated by the interaction of retinoids with specific nuclear receptors that belong to the steroid/thyroid/vitamin D receptor superfamily. Retinoid-X receptor (RXR) and retinoic acid receptor (RAR) mediated signaling is induced by retinoic acids (RA), which are involved in the regulation of skin permeability, differentiation, and immune response [7–9].

Glycolic acid also stimulates the growth of new skin. Although the exact mechanism of action of glycolic acid is still unknown,* alpha*-hydroxy acids decrease corneocyte cohesion and it has been suggested that this occurs by interference with the formation of ionic bonds. They dissolve adhesions between cells in the upper layers of the skin, inducing shedding of dry scales from the skin's surface, commonly referred to as exfoliation [2, 7].

Because retinoic acid and* alpha*-hydroxy acids are water soluble, creams and lotions of oil-in-water emulsions are usually the preferred choice. The most appropriate vehicle for a given product will depend on the purpose of the product and the patient's skin type. The vehicles may be hydro-alcohol-glycol solutions and gels (for oily and acneic skins), and creams and creamy lotions, ideal for dry and mature skins [7].

In addition to patient's skin type, it is essential to consider the influence of the vehicle on the effectiveness of a topical preparation. The vehicle may be the controlling factor in the release of the active ingredient from the formulation [10, 11]. The drug must leave the vehicle and enter the environment of the tissue before it can exert any biological activity. The release of drugs from various vehicles has been the subject of many reviews and research papers. Consistently, these papers indicate that a formulation or vehicle for a given chemical must be specifically designed for that chemical to obtain maximum drug release. Specific additives may enhance or retard release of a chemical from the vehicle; for example, lecithin improves the topical absorption of triamcinolone added in a poloxamer gel [12] and improves the topical absorption of vitamin A on a carbomer gel as well [13]. In addition, the composition of dermocosmetic formulations can influence the skin penetration of active ingredients and improve their efficacy on skin, as studied for epigallocatechin-3-gallate from green tea and vitamin A [10, 14].

Thus, the aim of this study was to compare the effects of retinoic and glycolic acid treatments on the hairless mouse epidermis thickness, horny layer renewal, and skin hydration, when added in gel, gel cream, or cream formulations.

## 2. Materials and Methods

### 2.1. Formulations Studied

The formulations consisted of a gel (HEC), a gel cream (HEC + hydrogenated lecithin), and a cream (ceteareth-20 + hydrogenated lecithin) with or without the addition of 6% glycolic acid (pH 3.5) or 0.05% retinoic acid (Table 1). The pH of all formulations was adjusted to 4.0.

### 2.2. Biological Assay

Adult male hairless mice (HRS/J-hairless, Jackson, Bar Harbor, ME) weighing on average 30 g were kept in individual cages and received commercial ration (Nuvilab CR-1), as well as water ad libitum. This study was carried out in accordance with the “Principles of Laboratory Animal Care” (NIH). The formulations gel, gel cream, and cream, with or without 6% glycolic acid or 0.05% retinoic acid, were applied in specific areas of the dorsum, once a day for 7 days.

### 2.3. Histology

After the application period, skin biopsies were obtained from the animals and semiserial 6 *μ*m thick sections were then stained with hematoxylin and eosin for general histopathological, morphometric, and stereologic analysis.

One week after starting the treatment, mice were euthanized by CO_2_ inhalation and skin fragments were obtained and immediately immersed in a fixing solution consisting of 85 mL of 80% alcohol, 10 mL formaldehyde, and 5 mL acetic acid. After 24 h the fixed fragments were dehydrated, cleared, and embedded in paraffin. Semiserial 6 mm thick sections were then obtained and each section corresponded to an interval of fifty sections; that is, ten sections were obtained from the 2 mm biopsy. The sections were stained with haematoxylin and eosin for general histopathological and histometric analysis [15, 16].

In the histopathological study, it was only possible to observe the qualitative alterations in the skin, after the use of the formulations.

### 2.4. Morphometry

For the morphometric study (analysis of the nucleus of cells from the epithelial layers), the skin sections obtained from each experimental group were analyzed with a Henamed light microscope equipped with a 100x immersion objective and a light camera (Jena). The largest and smallest diameters of the nuclei of the cells from the basal and spinous layers of the epidermis were measured and the mean diameter and nuclear volume were estimated. The following karyometric parameters were estimated.

- *Mean diameter M* = (*D* · *d*)^1/2^.
- *Volume V* = 6^−1^ · *π* · *M* ^3^.

### 2.5. Stereology

In the stereologic study, which is a quantitative evaluation, the epithelial thickness, the thickness of each layer of the epidermis, the numerical nuclear density, and the cytoplasmic and cell volume were obtained. A grid idealized by Merz printed on paper (Figure 1) was used to draw the epithelial structures [2] to use the stereologic equation with respect to the parameter studied using GMC program.

The Merz grid was used to count points on a given histological structure and also to count intersections between two contiguous structures, by considering the number of points that fall on the structure under study in the former case and the number of times that neighboring surfaces cut the curved line in the latter.

Thus, in order to obtain the thickness, the numerical nuclear density, and the cytoplasm volume, we used point counting (2000 per animal, corresponding to the product of 20 microscope fields per 100 points on the grid) or the number of intersections, according to the requirements of the stereologic equation with respect to the parameter studied.

*Numerical Nuclear Density (Nvn)*. The area of the epithelium within the test system was evaluated by counting the points that fall on it, and the epithelial volume was proportional to it. The nuclei inside the standard square were then counted. The total area of the square is 50.625 *μ*m^2^ in two fields per section, for a total of 20 fields per block and this permits to obtain the number of nuclear sections of the area (Nav). The number of nuclei per unit volume (numerical nuclear density, Nvn) was calculated using the following equation:

(1) $$\begin{array}{c} \text{Nvn}=\frac{\text{Nav}}{D+T}, \end{array}$$

where *D* is the mean nuclear diameter previously estimated by karyometry and *t* is the thickness of the section (6 *μ*m). The result obtained corresponds to the number of nuclei per mm^3^.

*Cytoplasmic Volume and Epithelial Cell Volume*. Cytoplasmic volume (*V*_ct_) was estimated from the previously determined nuclear volume and the corrected nucleus/cytoplasm ration. In turn, the sum of the mean nuclear and cytoplasmic volumes provides the estimated value of the epithelial cell. The cytoplasmic volume is given by the following ratio:

(2) $$\begin{array}{c} V_{\text{ct}}=\frac{V_{n}}{\text{corrected}\cdot n/c}. \end{array}$$

The volume of the epithelial cell, in turn, is given by the following equation:

(3) $$\begin{array}{c} V_{\text{cela}}=V_{n}+V_{\text{ct}}. \end{array}$$

*Mean Epithelial Thickness*. Mean epithelial thickness was estimated by the formula of Weibel [12, 13]:

(4) $$\begin{array}{c} E=\frac{P\cdot L}{2\left(I_{K}+I_{\text{ct}}\right)}, \end{array}$$

where *P* is the number of points that fell on the epithelium, *L* is the length of the test line, and *I*_*K*_ and *I*_ct_ are the numbers of intersections of the test line with the epithelium-keratin interface and the epithelium-connective tissue interface, respectively.

### 2.6. Statistical Analysis

Morphometric and stereologic data were analyzed statistically using analysis of variance, a parametric test, followed by Tukey test.

## 3. Results and Discussion

The results obtained in this investigation are shown in Figures 2 to 6.

### 3.1. Histology

The areas treated with gel cream or cream (Figures 2(d) and 2(g)) presented an enhancement on the epidermis thickness, with the basal cells and their nuclei being more voluminous, when compared to gel treatment (Figure 2(a)). An enhancement in the nuclear volume in the spinous and basal layers could also be observed.

When retinoic acid was present in the formulations studied, the epidermis thickness was greatly increased, and the basal layer showed both cells and nuclei increased. In addition, the effects observed from retinoic acid topical use occurred independently from vehicles studied (Figures 2(b), 2(e), and 2(h)). There was an apparent increase of the dermal thickness when compared to the vehicles (formulations without retinoic acid).

Glycolic acid increased the epidermis thickness and also the cell volume, when it was present in the cream formulation. Glycolic acid effects were vehicle dependent because better results were obtained only when this active substance was added in the gel cream and cream formulations (Figures 2(c), 2(f), and 2(i)).

### 3.2. Morphometry and Stereology

The statistical analysis results of the nuclear volume obtained in the morphometric study and the cell volume and epithelial and horny layer thickness obtained in the stereologic evaluation are shown in Figures 3 to 7.

Both glycolic acid and retinoic acid acted on the epidermis. However, this fact has occurred in different intensity and way, depending upon the variable studied. Retinoic acid enhanced the epithelial thickness (*P* < 0.001) (Figure 3) (G: 25.27 ± 2.16, GC: 25.07 ± 1.75, and C: 27.19 ± 0.42 *μ*m), which can suggest that epidermal cells are in intense renewal process, which was also observed by other authors who studied retinol effects on the skin [17, 18]. On the other hand, glycolic acid reduced this thickness (*P* < 0.001) (Figure 3) (G: 20.12 ± 3.20, GC: 18.24 ± 2.60, and C: 19.01 ± 1.18 *μ*m). Rodrigues and Maia Campos [2] observed that a 15-day treatment of hairless mouse skin with glycolic acid enhanced the epithelium thickness; consequently the formulation of the present study could be suggested, since a lower concentration of this acid and a higher pH as well as the period of application were not enough to provoke a statistically significant enhancement of epithelium thickness.

The effect provoked by retinoic acid in the horny layer renewal (Figure 7) was higher than the glycolic acid effect, since retinoic acid caused a reduction in the horny layer thickness (*P* < 0.05) (retinoic acid: G: 7.70 ± 0.85, GC: 7.22 ± 1.30, and C: 8.87 ± 0.91; glycolic acid: G: 15.43 ± 2.08, GC: 7.00 ± 0.66, and C: 8.79 ± 4.92), which can be due to higher cellular renewal stimulation and a higher desquamation ratio. This enhancement of epithelium thickness and reduction of horny layer thickness were also reported by Zouboulis [19].

Glycolic acid, after a 7-day treatment, only reduced the granular layer thickness (Figure 4) which suggested that the exfoliation process was only beginning.

Retinoic acid produced a significant increase in the thickness of the basal, spinous, and granular layers (*P* < 0.01) (retinoic acid: basal: 8.55, spinous: 7.52, and granular: 4.7 *μ*m; vehicle: basal: 7.3, spinous: 5.6, and granular: 2.9 *μ*m) (Figure 4) without the enhancement of the number of cells (*P* < 0.001) (basal: 1.9, spinous: 1.6, and granular: 1.7 cells × 10^5^/mm^3^), probably due to the extracellular hydration. No inflammation was evident.

Summers et al. [20] reported that epidermis cell renewal process usually leads to the formation of a thicker horny layer (hyperkeratinization) or sometimes to a thinner horny layer, which depends on the corneocyte cohesion.

Retinoic acid treatment provoked an enhancement of epithelial layers thickness (basal, spinous, and granular layers), when compared to formulations with and without glycolic acid.

Retinoic acid also provoked the enhancement of nuclear and cell volumes (*P* < 0.001) (Figures 5 and 6), one of the reasons that cause the epithelium thickening (Figure 3). This way, it could be suggested that the enhancement of epithelium thickness occurred due to an enhancement of the intracellular hydration. Glycolic acid, except in granular layer, has not modified epithelial layers thickness significantly (Figure 4).

It can be suggested that intra- and extracellular edema (hydration) is a possible cause of the enhancement of epithelium thickness since Maia Campos et al. [15] and Silva and Maia Campos [16] also described these effects in guinea pig skin with the application of other active substances.

The alterations observed in the cell nuclei can suggest an alteration on their functionality and could reflect an enhancement of nuclei activity [16].

The enhancement of nuclear volume provoked by the retinoic acid treatment was connected with the enhancement of cytoplasm and cell volume, which confirms the presence of intracellular edema. On the other hand, glycolic acid did not alter significantly the cytoplasm and cellular volume when compared to the vehicle (formulation without active substances).

The results obtained showed that one of the benefits from the use of these acids in dermocosmetic formulations is caused by the hydration of the epidermis.

It is also important to highlight that, under the experimental conditions, retinoic acid effects are independent from the vehicle and, consequently, dermatologists could choose any of the studied vehicles (gel, gel cream, and cream) according to skin types that its antiaging effects will not be altered.

Despite the fact that hairless mouse epidermis thickness is similar to human, differences between hairless mouse and human skin mean that caution is needed in interpreting the results. Nevertheless, the results obtained in this research contributed to orient and elucidate the possible effects of these acids on the epidermis.

## 4. Conclusion

Under the present experimental conditions, we concluded the following.

- The effects of retinoic acid were independent from the vehicle because the evaluated variables were not different when this substance was added to gel, gel cream, and cream. The glycolic acid effects were dependent on the vehicles since it caused better results when added to cream and gel cream.
- Retinoic acid was more effective when compared to glycolic acid, mainly in the cell renewal (due to the enhancement of nuclear volume) and the exfoliation process because it decreased the horny layer thickness.
- Retinoic acid was indicated to improve the skin conditions, in a short time application period, due to the horny layer renewal effect.

## Figures and Tables

**Figure 1:** The Merz grid.

**Figure 2:** Photomicrographs of hairless mice skin. Magnification: ×960, HE. Yellow stars represent nuclei of the basal cells and red rectangles represent spinous layers.

**Figure 3:** Mean values of epithelial thickness obtained by the treatment with the active substances in different formulations (ANOVA, *n* = 5 measurements, mean ± SEM).  ^*^Significantly different from the vehicle treated area (*P* < 0.001).

**Figure 4:** Mean values of epithelial layers thickness obtained by the treatment with the active substances in different formulations (ANOVA, *n* = 5 measurements, mean ± SEM).  ^*^Significantly different from the vehicle treated area (*P* < 0.01).

**Figure 5:** Mean values of nuclear volume obtained by the treatment with the active substances in different formulations (ANOVA, *n* = 5 measurements, mean ± SEM).  ^*^Significantly different from the vehicle treated area (*P* < 0.001).

**Figure 6:** Mean values of cell volume obtained by the treatment with the active substances in different formulations (ANOVA, *n* = 5 measurements, mean ± SEM).  ^*^Significantly different from the vehicle treated area (*P* < 0.001).

**Figure 7:** Mean values of horny layer thickness obtained by the treatment with the active substances in different formulations (ANOVA, *n* = 5 measurements, mean ± SEM).  ^*^Significantly different from the vehicle treated area (*P* < 0.05).

**Table 1:** Formulations studied.

	Percentage of components in each formulation (w/w)		
	Gel	Gel cream	Cream
Hydroxyethylcellulose	2.00	2.00	
Hydrogenated lecithin	—	1.00	1.00
Cetearyl alcohol and ceteareth-20	—	—	4.00
Glycerin	3.00	3.00	3.00
Squalane	2.00	2.00	2.00
Butylated hydroxytoluene	0.05	0.05	0.05
Methyldibromo-glutaronitrile and phenoxyethanol	0.20	0.20	0.20
Propylene glycol	2.00	2.00	2.00
Distilled water to.	100.00	100.00	100.00

## References

[1] Orfanos C. E., Zouboulis C. C., Almond-Roesler B., Geilen C. C. (1997). Current use and future potential role of retinoids in dermatology. *Drugs*.

[2] Rodrigues L. H. T., Maia Campos P. M. B. G. (2002). Comparative study of the effects of cosmetic formulations with or without hydroxy acids on hairless mouse epidermis by histopathologic, morphometric, and stereologic evaluation. *Journal of Cosmetic Science*.

[3] Sadick N. S., Karcher C., Palmisano L. (2009). Cosmetic dermatology of the aging face. *Clinics in Dermatology*.

[4] Davis E. C., Callender V. D. (2011). Aesthetic dermatology for aging ethnic skin. *Dermatologic Surgery*.

[5] Kakudo N., Kushida S., Suzuki K., Kusumoto K. (2013). Effects of glycolic acid chemical peeling on facial pigment deposition: evaluation using novel computer analysis of digital-camera-captured images. *Journal of Cosmetic Dermatology*.

[6] Kligman L. H., Sapadin A. N., Schwartz E. (1996). Peeling agents and irritants, unlike tretinoin, do not stimulate collagen synthesis in the photoaged hairless mouse. *Archives of Dermatological Research*.

[7] Ramos-e-Silva M., Hexsel D. M., Rutowitsch M. S., Zechmeister M. (2001). Hydroxy acids and retinoids in cosmetics. *Clinics in Dermatology*.

[8] Michel S., Jomard A., Démarchez M. (1998). Pharmacology of adapalene. *The British Journal of Dermatology*.

[9] Mihály J., Gericke J., Aydemir G. (2012). Reduced retinoid signaling in the skin after systemic retinoid-X receptor ligand treatment in mice with potential relevance for skin disorders. *Dermatology*.

[10] Gianeti M. D., Wagemaker T. A. L., Seixas V. C., Maia Campos P. M. B. G. (2012). The use of nanotechnology in cosmetic formulations: the influence of vehicle in the vitamin A skin penetration. *Current Nanoscience*.

[11] Bagatin E., Wagemaker T. A. L., Aguiar N. R. (2014). Tretinoin-based formulations—influence of concentration and vehicles on skin penetration. *Brazilian Journal of Pharmaceutical Science*.

[12] Bentley M. V. L. B., Marchetti J. M., Ricardo N., Ali-Abi Z., Collett J. H. (1999). Influence of lecithin on some physical chemical properties of poloxamer gels: rheological, microscopic and in vitro permeation studies. *International Journal of Pharmaceutics*.

[13] Maia Campos P. M. B. G., Benetton S. A., Eccleston G. M. (1998). Vitamin A skin penetration—studies of some vehicles currently used. *Cosmetics & Toiletries*.

[14] Dal Belo S. E., Gaspar L. R., Maia Campos P. M. B. G., Marty J.-P. (2009). Skin penetration of epigallocatechin-3-gallate and quercetin from green tea and *Ginkgo biloba* extracts vehiculated in cosmetic formulations. *Skin Pharmacology and Physiology*.

[15] Maia Campos P. M. B. G., Ricci G., Semprini M., Lopes R. A. (1999). Histopathological, morphometric, and stereologic studies of dermocosmetic skin formulations containing vitamin A and/or glycolic acid. *Journal of Cosmetic Science*.

[16] Silva G. M., Maia Campos P. M. B. G. (2000). Histopathological, morphometric and stereological studies of ascorbic acid and magnesium ascorbyl phosphate in a skin care formulation. *International Journal of Cosmetic Science*.

[17] Kang S., Duell E. A., Fisher G. J. (1995). Application of retinol to human skin *in vivo* induces epidermal hyperplasia and cellular retinoid binding proteins characteristic of retinoic acid but without measurable retinoic acid levels or irritation. *Journal of Investigative Dermatology*.

[18] Förster T., Jassoy C., Petersohn D. Investigating the influence of a retinol cream on the skin.

[19] Zouboulis C. C. (2000). Retinoids: is there a new approach?. *IFSCC Magazine*.

[20] Summers R. S., Summers B., Chandar P., Feinberg C., Gursky R., Rawlings A. V. (1996). The effect of lipids, with and without humectant, on skin xerosis. *Journal of Cosmetic Science*.

